# Peak exercise capacity prediction from a submaximal exercise test in coronary artery disease patients

**DOI:** 10.3389/fphys.2013.00243

**Published:** 2013-09-04

**Authors:** Arto J. Hautala, Antti M. Kiviniemi, Jaana J. Karjalainen, Olli-Pekka Piira, Samuli Lepojärvi, Timo Mäkikallio, Heikki V. Huikuri, Mikko P. Tulppo

**Affiliations:** ^1^Department of Exercise and Medical Physiology, Verve ResearchOulu, Finland; ^2^Department of Internal Medicine, Institute of Clinical Medicine, University of OuluOulu, Finland

**Keywords:** exercise capacity, rating of perceived exertion, exercise testing, cardiac patients, prediction

## Abstract

The purpose of this study was to determine whether a rating of perceived exertion scale (RPE) obtained during submaximal exercise could be used to predict peak exercise capacity (MET_peak_) in coronary artery disease (CAD) patients. Angiographically documented CAD patients (*n* = 124, 87% on β blockade) completed a symptom-limited peak exercise test on a bicycle ergometer, reporting RPE values at every second load on a scale of 6–20. Regression analysis was used to develop equations for predicting MET_peak_. We found that submaximal METs at a workload of 60/75 W (for women and men, respectively) and the corresponding RPE (METs/RPE ratio) was the most powerful predictor of MET_peak_ (*r* = 0.67, *p* < 0.0001). The final model included the submaximal METs/RPE ratio, body mass index (BMI), sex, resting heart rate, smoking history, age, and use of a β blockade (*r* = 0.86, *p* < 0.0001, SEE 0.98 METs). These data suggest that RPE at submaximal exercise intensity is related to MET_peak_ in CAD patients. The model based on easily measured variables at rest and during “warm-up” exercise can reasonably predict absolute MET_peak_ in patients with CAD.

## Introduction

A large volume of data confirms the inverse dose–response relationship between peak exercise capacity (MET_peak_) and all-cause mortality in both male and female coronary artery disease (CAD) patients irrespective of the use of β-blocking medication (Kavanagh et al., 2002, 2003), including patients with a history of myocardial infarction, coronary artery bypass grafting (CABG), percutaneous coronary intervention (PCI), and chronic heart failure (Perk et al., 2012). Although being able to measure MET_peak_ by the “golden standard” method of a direct incremental symptom-limited peak exercise test, it may not be feasible in everyday clinical settings for rehabilitation or in assessment of functional capacity in CAD patients. Due to increasing constraints of time, equipment, patient safety and personnel needed to carry out these tests, practical applications are typically submaximal laboratory or field tests; e.g., a six-minute walking test (Lipkin et al., 1986) is recommended for CAD patients (Wijns et al., 2010). However, several adequate submaximal tests that estimate MET_peak_ are based on nomograms which predict MET_peak_, assuming a more or less linear increase in heart rate simultaneously with increasing workload and oxygen uptake (Astrand and Ryhming, 1954; WHO, 1968). These tests are able to predict MET_peak_ in healthy subjects but not in CAD patients due to the use of medication, particularly β blockades. Therefore, accurate predictive estimates for MET_peak_ in CAD patients are warranted.

The ratings of perceived exertion (RPE) scale (Eston and Williams, 1988) is widely accepted for obtaining a subjective estimate of work intensity and as a means of quantifying, monitoring, and evaluating exercise intensity not only in healthy subjects, but also in CAD patients (Pollock and Pels, 1984; Corra et al., 2010; Scherr et al., 2013). The practical use of RPE for exercise prescription also in patients with β blockades is well documented (Eston and Connolly, 1996; Goss et al., 2011). Therefore, we hypothesized that RPE during submaximal exercise can be used to predict MET_peak_ in CAD patients. The purpose of this study was firstly to develop an equation for predicting MET_peak_ using assessment of RPE during submaximal exercise in CAD patients, and secondly to validate the developed model and estimate the reproducibility of the model in an independent sample of CAD patients.

## Materials and methods

The patients in the test group (*n* = 124, 27 women) belong to a larger Innovation to Reduce Cardiovascular Complications of Diabetes at the Intersection study (ARTEMIS) taking place in the Division of Cardiology at Oulu University Hospital (Oulu, Finland) and the Department of Exercise and Medical Physiology at Verve (Oulu, Finland). The ARTEMIS study is registered at ClinicalTrials.gov, Record 1539/31/06. In addition, we recruited from Oulu University Hospital an independent sample of volunteer CAD patients who had suffered acute coronary syndrome to serve as the validation group (*n* = 42, 12 women) and to test the developed equation as a predictor of MET_peak_. The patients in the validation group belong to a larger Effectiveness of Exercise Cardiac Rehabilitation study (EFEX-CARE) taking also place in the above mentioned institutions. The EFEX-CARE study is registered at ClinicalTrials.gov, Record NCT01916525. Demographic characteristics of the study population are presented in Table 1. The subjects were not allowed to eat or to drink coffee for 3 h before the tests. Strenuous physical activity and alcohol consumption were prohibited on the day of the tests and the preceding day. The study was performed according to the Declaration of Helsinki, the local research ethics committee of the Northern Ostrobothnia Hospital District approved the protocol, and all the subjects gave their written informed consent.

**Table 1:** **Demographic characteristics of study populations**.

	**Test, *n* = 124**	**Validation, *n* = 42**	***p*-value**
Patients with T2D	69 (56%)	11 (26%)	0.001
Sex (M/F)	97 (78%)/27 (22%)	30 (71%)/12 (29%)	0.402
Age, years	62 ± 5	60 ± 10	0.105
Height, m	1.71 ± 0.8	1.70 ± 0.9	0.668
Weight, kg	83 ± 15	81 ± 18	0.435
BMI, kg/m^2^	28.3 ± 4.1	27.7 ± 4.6	0.391
Waist-hip ratio	0.99 ± 0.11	0.99 ± 0.15	0.924
Systolic BP, mmHg	146 ± 21	138 ± 22	0.040
Diastolic BP, mmHg	80 ± 10	76 ± 9	0.053
Current smokers	13 (10%)	8 (19%)	0.180
Depression score	5.0 ± 5.0	5.3 ± 5.4	0.755
**HISTORY OF AMI**			
NSTEMI	40 (32%)	19 (45%)	0.262
STEMI	24 (19%)	11 (26%)	0.384
**REVASCULARIZATION**			
PCI	73 (59%)	32 (76%)	0.063
CABG	27 (22%)	2 (5%)	0.010
**CARDIAC FUNCTION**			
LVEF, %	66 ± 8	65 ± 7	0.366
LVMI	101 ± 23	102 ± 23	0.804
CCS class	1.2 ± 0.4	1.3 ± 0.5	0.237
**PEAK EXERCISE TEST**			
Rest HR, bpm	59 ± 9	60 ± 8	0.700
Peak HR, bpm	130 ± 19	132 *±* 19	0.665
Peak METs	7.1 ± 1.9	7.1 ± 2.0	0.941
Estimated peak mets	7.2 ± 1.6	7.2 ± 1.7	0.788
**LABORATORY ANALYSES**			
HbA1c, %	6.3 ± 0.8	6.1 ± 1.1	0.151
Fasting plasma glucose, mmol/l	6.3 ± 1.4	5.7 ± 1.1	0.021
Total cholesterol, mmol/l	4.0 ± 0.8	4.0 ± 0.9	0.609
HDL cholesterol, mmol/l	1.2 ± 0.3	1.3 ± 0.3	0.731
LDL cholesterol, mmol/l	2.3 ± 0.6	2.4 ± 0.8	0.154
Triglycerides, mmol/l	1.5 ± 0.9	1.5 ± 0.7	0.999
**MEDICATION**			
Oral antidiabetics	57 (46%)	10 (24%)	0.012
Insulin	10 (8%)	4 (10%)	0.755
Beta blockers	108 (87%)	35 (83%)	0.606
ACEI/ARB	74 (60%)	30 (71%)	0.200
Lipid lowering drugs	114 (92%)	40 (95%)	0.732
Anticoagulants	121 (98%)	41 (98%)	0.989
Calcium antagonists	26 (21%)	7 (17%)	0.658
Nitrates	29 (23%)	11 (26%)	0.683
Diuretics	38 (31%)	8 (19%)	0.167

All the patients were diagnosed as having CAD, which had been documented previously by coronary angiography. In recruiting the CAD patients, the following exclusion criteria were adhered: advanced age (>75 years), body mass index (BMI) >40 kg/m^2^, NYHA class III or IV, left ventricular ejection fraction (LVEF) <40%, scheduled cardiac revascularization therapy, unstable angina pectoris, severe peripheral atherosclerosis, or inability to perform an exercise stress test, e.g., due to musculoskeletal problems. Type 2 diabetes (T2D) was verified according to the current criteria (Spies et al., 2005). Left ventricular systolic function was assessed using 2-D echocardiography (Vivid 7, GE Healthcare, Wauwatosa, WI, USA). Blood samples were obtained for analysis of blood lipids, plasma glucose, and glycated hemoglobin (HbA1c) levels (Oulu University Hospital, Oulu, Finland).

The following protocol was performed in the Department of Exercise and Medical Physiology at Verve (Oulu, Finland). Blood pressure was measured (average of two measurements) in a supine position after a 10-min resting period (Tango, Sun-Tech, Raleigh, NC, USA). The patients performed an incremental symptom-limited peak exercise test on a bicycle ergometer (Monark Ergomedic 839 E, Monark Exercise AB, Vansbro, Sweden) for assessment of MET_peak_. MET_peak_ was used as an outcome of maximal exercise capacity, since measurement of peak oxygen consumption is not applied as daily routine in hospital. One metabolic equivalent (MET) is the rate of energy expenditure at rest (approximately 1 kcal per kilogram of body weight per hour), which equates to oxygen consumption approximately 3.5 ml/kg of body weight per minute for an average adult (Jette et al., 1990). The test was started at 30 Watts (W) and the work rate was increased by 15 W in men and 10 W in women every minute until voluntary exhaustion or ST segment depression >0.2 mV in electrocardiography (ECG). Prior to performing the exercise test, the RPE scale was explained to each participant by trained practitioners (Borg, 1982). RPE values were asked in the 15 s before the end of every second workload on a scale of 6–20 (Borg, 1970). MET_peak_ was calculated from the mean workload during the last minute of the test. A 15-lead ECG (GE Healthcare, CAM-14, Freiburg, Germany) was taken when the patients sat 1 min on a bicycle without speaking, during the exercise and 10 min after the exercise in a supine position.

After the predictive model was developed, we applied the equation to a seven-minute submaximal testing procedure with a bicycle (Monark 939E, Monark Exercise AB, Vansbro, Sweden). Then we requested the patients in the validation group to visit our laboratory at Verve 1 day before the measurement of MET_peak_ to perform a seven-minute submaximal test. Furthermore, we asked the same patients to visit our laboratory 1 week after the initial visit to perform submaximal test again to assess the reproducibility of test. In the laboratory, first the patients sat 1 min on a bicycle without speaking and their average resting heart rate (Polar Electro, Kempele, Finland) was measured and recorded on a Smart Card (HUR Oy, Kokkola, Finland). Then they started cycling at 30 W for women and 50 W for men. As during MET_peak_ testing, the RPE scale was explained to each participant. In the 15 s before the end of every one-minute workload the RPE value was asked on a scale of 6–20 and recorded on the Smart Card. Based on the reported RPE after each minute, workload was automatically adjusted so that the given RPE value would be 13 at the end of 5 min of cycling. For example, if RPE after the first minute was 12, the second workload increased automatically by 5 W to have an RPE of 13 after the second minute. Finally, after the 5-minute “warm up,” the patients sat one more minute on the bicycle without speaking and their average recovery heart rate was measured and recorded on the Smart Card. Then the collected data were uploaded to a computer for calculation of predicted MET_peak_ (HUR Smart Card Software, HUR Oy, Kokkola, Finland).

Data normality was confirmed with the Kolmogorov-Smirnov goodness-of-fit test. Differences between the test and validation groups were analyzed by using independent-samples *t* tests and chi-square tests. The data from the MET_peak_ test were used to develop equations for estimating MET_peak_ using stepwise linear regression analysis. All the significant demographic, medication, laboratory, leisure-time physical activity collected with the questionnaire and echocardiographic variables from Spearman's correlation analyses and *t* tests were included in the linear regression analyses if their *p*-values were <0.05 to find the predictors that maximized the *R*-value. The following parameters were used to yield the best predictive equation: age, sex, BMI, hip and waist size, smoking history, use of β blockade, T2D, heart rate before cycling, and submaximal METs at a workload of 60/75 W (for women and men, respectively) and corresponding RPE (METs/RPE ratio). The METs/RPE ratio was defined considering body weight and resting energy expenditure as follows: [(60/75 W × 12 + 3.5 × body weight)/(3.5 × body weight)] (Adams, 1990; ACSM, 1995).

The prediction of MET_peak_ was compared with the measured MET_peak_ in both the test and validation groups using linear regression analysis and standard error of the estimate (SEE). A Bland-Altman analysis of measurement differences plotted against mean values was used to assess the degree of agreement (Bland and Altman, 1986) and to estimate the reproducibility of the developed submaximal test. The statistical analyses were performed using SPSS software, version 19.0 (SPSS Inc., Chicago, USA). A *p*-value <0.05 was considered statistically significant.

## Results

Table 1 presents the demographic characteristics as well as the measured and estimated MET_peak_ values in both populations. The groups did not differ in measured or estimated measured MET_peak_. There were more T2D patients, higher systolic blood pressure, and more revascularization by CABG in the test group than in the validation group (*p* = 0.001, *p* = 0.040, and *p* = 0.010, respectively). Accordingly, fasting plasma glucose was higher and there were more oral antidiabetic users in the test group than in the validation group (*p* = 0.021 and *p* = 0.012, respectively).

During the measurement of MET_peak_ in the test group, submaximal METs at a workload of 60/75 W (55 ± 15% of measured W_peak_) was 4.0 ± 0.5 (59 ± 12% of measured MET_peak_) and the corresponding RPE was 11.8 ± 2.1. The submaximal METs/RPE ratio was the most powerful predictor of MET_peak_ (*r* = 0.67, *p* < 0.0001) explaining 44% of the variability in MET_peak_. The final stepwise regression model correlated strongly with that of MET_peak_ after including the parameters in the following order: submaximal METs/RPE ratio, BMI, sex, heart rate before cycling, smoking history, age, and use of β blockade (*r* = 0.86, SEE 0.98 METs, *p* < 0.0001, Figure 1A). The following best predictive equation explained 74% of the variability in MET_peak_: 16.047 + 6.227 (submaximal/RPE ratio) − 0.178 (BMI) + 1.412 (sex) − 0.057 (heart rate before cycling) − 0.603 (smoking history) − 0.048 (age) − 0.605 (use of β blockade). The mean difference between actual and predicted MET_peak_ was 0.09 ± 1.00 METs. The Bland-Altman plot found 94% of the data points within the limits of agreement in the test group (Figure 2A).

**Figure 1:** **Regression between predicted peak exercise capacity (MET_peak_) and measured from the test (A) and validation (B) groups of coronary artery disease patients**.

**Figure 2:** **Bland-Altman plot for predicted and measured MET_peak_ in both test (A) and validation (B) groups**. The bold black lines indicate the mean difference between measured and predicted MET_peak_ and the bold gray lines indicate the 95% limits of agreement (±2 SD).

MET_peak_ values collected from the seven-minute submaximal testing procedure showed a strong association with the measured MET_peak_ (*r* = 0.77, *p* < 0.0001, SEE 1.38 METs, Figure 1B). The mean difference between actual and predicted MET_peak_ was 0.04 ± 1.37 METs. In the validation group, 98% of the data points fell within the limits of agreement (Figure 2B). The difference among two measurements of METs in the case of 26 patients, who were able to participate the reproducibility study, are plotted as a function of each subject's mean value (*r* = 0.98, *p* < 0.0001, SEE 0.38 METs, Figure 3).

**Figure 3:** **Differences among two measurements performed on each of 26 patients as a function of their mean values for METs**.

## Discussion

This study showed that RPE at submaximal exercise intensity is related to measured MET_peak_ in CAD patients. The data support the view that a regression model based on easily measured variables at rest and during “warm-up” exercise can be used to predict MET_peak_ in patients with CAD in whom a peak exercise test may not be feasible, and in repeated assessments of exercise capacity after therapeutic interventions, e.g., during rehabilitation programs, even on a weekly or monthly basis.

Borg's RPE scale is a widely used psycho-physical tool for subjectively assessing work intensity during exercise. It is also well documented that the RPE scale can be used to increase the accuracy of monitoring and the prescription of exercise intensity in the cardiac population using β blockade therapy (Pollock and Pels, 1984; Eston and Connolly, 1996; Goss et al., 2011). In the present study we found that a submaximal METs/RPE ratio where an RPE value of approximately 12 was reached at an intensity of 60/75 W was associated most strongly with the measured MET_peak_. We decided to use a target RPE of 13 at the end of 5 min of cycling in the developed submaximal testing procedure because it is well in line with the finding that an RPE of 14 might indicate fatigue if an incremental treadmill test is continued in CAD patients using β blockades (Goss et al., 2011). Furthermore, according to the latest study by Scherr et al., training intensities corresponding to an RPE range of 11–13 (“fairly light” to “somewhat hard”) should be recommended for CAD patients (Scherr et al., 2013). Since safety during exercise testing is very important, we feel the developed and validated submaximal test in this study meets these demands appropriately, as well.

A 6-min walking test is a much-used, safe, and well-tolerated method for assessing exercise capacity in cardiac patients (Gayda et al., 2004; Wijns et al., 2010) and it also has prognostic value in predicting cardiovascular events in CAD patients (Beatty et al., 2012; Cacciatore et al., 2012). When the results of the walking test are compared with measured peak exercise capacity expressed as peak oxygen consumption in cardiac patients, the correlation values have varied from 0.58 to 0.69, giving an SEE normalized by mean peak oxygen consumption from 21 to 28% (Cahalin et al., 1996; Faggiano et al., 1997; Zugck et al., 2000; Opasich et al., 2001). In the present study, we found that the developed submaximal exercise test correlated from 0.77 to 0.86 with the measured MET_peak_, indicating an SEE from 14 to 19%. Bland-Altman analysis showed that only a few values fell outside the 95% limits of agreement, which suggests a good agreement between the actual and estimated MET_peak_ values. Furthermore, repeated tests performed for the validation group showed that developed test model is highly reproducible, which emphasize the use of this test as an individual monitoring tool for exercise capacity. Taken together, the present data support the concept that the estimated MET_peak_ values obtained from a submaximal exercise test are sufficiently accurate, as they provide also an excellent fit with published results.

It should be noted that the test and validation groups differed from each other in certain demographic characteristics, e.g., there were more revascularizations by CABG and a greater tendency toward higher blood pressure in the test group than in the validation group. Potentially, the differences are explained by the fact that there was more T2D in the test group. The patients in the test group belong to a larger ARTEMIS study, where the aim is to gather two groups of patients; CAD patients with and without T2D. The patients in the separate validation group were volunteers who had suffered from acute coronary syndrome. However, T2D was not related to measured MET_peak_ and it was not included in the predictive equation. Still, it remains speculative if the minor discrepancy in the accuracy of the test between groups (SEE 14 vs. 19%) is partly explained either by the differences in demographic parameters or the implemented submaximal testing procedure or both.

Based on the findings of the present study, the proposed submaximal testing procedure can be useful for CAD patients also in terms of motivation for physical activity and exercise training, since the assessment of MET_peak_ is available during the “warm-up” of a single exercise session and no extra time for exercise testing is needed. However, the ability of our test to follow changes in MET_peak_ during rehabilitation needs to be confirmed in further studies. Another advantage of the developed test is the use of guided self-regulated moderate exercise intensity expressed as target RPE 13 at the end of the “warm up.” In this regard, a certain learning effect of subjective feeling of moderate-intensity exercise could be used to facilitate a transition from a supervised to a self-guided exercise program and hopefully to serve as a contributing factor for better adherence to a physical activity program. Finally, almost all of the patients in our study were under continued β-blocking medication, and cessation of β blockades usually is not possible during exercise tests. Therefore, our results are valid and could be generalized in clinical practice in CAD patients who are under continued β-blocking medication.

In conclusion, the current study shows that Borg's RPE is a practical tool for assessing MET_peak_ in secondary preventive medicine. RPE at submaximal exercise intensity is related to absolute MET_peak_ in CAD patients. The data reveal that the relationships between RPE and exercise intensity together with easily measured variables at rest and during “warm-up” exercise can reasonably predict MET_peak_ in patients with CAD.

### Conflict of interest statement

The authors declare that the research was conducted in the absence of any commercial or financial relationships that could be construed as a potential conflict of interest.

## Abbreviations

ACEI: angiotensin conversion enzymes inhibitor
AMI: acute myocardial infarction
ARB: angiotensin receptor blocker
ACEI/ARB: patients using at least one of them
BMI: body mass index
BP: blood pressure
CABG: coronary artery bypass grafting
CCS: Canadian Cardiovascular Society angina classification
HbA1c: glycated hemoglobin
HDL: high-density lipoprotein
HR: heart rate
LDL: low-density lipoprotein
LVEF: left ventricular ejection fraction
LVMI: left ventricular mass index
METs: metabolic equivalents
n: number of subjects
NSTEMI: non-ST segment elevation myocardial infarction
PCI: percutaneous coronary intervention
T2D: type 2 diabetes
STEMI: ST segment elevation myocardial infarction.
